# Association between Dietary Pattern, Nutritional Status, Metabolic Factors, and Nonalcoholic Fatty Liver Disease

**DOI:** 10.1155/2022/4157403

**Published:** 2022-08-02

**Authors:** Guisheng Xing, Ying Huang, Xiao Liu

**Affiliations:** ^1^Department of Medical Affairs, Ningbo Zhenhai People's Hospital (Ningbo No. 7 Hospital), Ningbo, Zhejiang 315200, China; ^2^Clinical Laboratory, Ningbo Zhenhai People's Hospital (Ningbo No. 7 Hospital), Ningbo, Zhejiang 315200, China; ^3^Department of Gastroenterology, Ningbo Zhenhai People's Hospital (Ningbo No. 7 Hospital), Ningbo, Zhejiang 315200, China

## Abstract

Nonalcoholic fatty liver disease (NAFLD) can be harmful to the body to varying degrees, and over a prolonged period, patients may develop steatotic cirrhosis or even develop liver cancer based on cirrhosis. Moreover, its harms are related to its severity. Patients with severe steatosis develop hepatocyte destruction, transaminase abnormalities, and long-term progression to steatotic cirrhosis, or even liver cancer, which should be treated aggressively. In order to provide theoretical basis for the prevention and early intervention of NAFLD, we analysis the relationship between nonalcoholic fatty liver disease(NAFLD) and dietary pattern, nutritional status, metabolic factor A total of 517 participants (200 males and 317 females) recruited in this study were gained from the health check center of The Ningbo Seventh Hospital, Ningbo, China, from September 2018 to August 2019. Patients diagnosed with NAFLD were selected as the study subjects. The data on the dietary pattern, nutritional status, and metabolic factors were collected for further analysis. A total of 517 eligible participants (317 females and 200 males) were involved in this study, with a mean age of 54.7 ± 16.7 years. Dessert and fruit diet, healthy dietary pattern, animal food dietary pattern, high salt diet mode, triglyceride, uric acid, adiponectin, and waist-hip ratio were significantly different between the two groups (*P* < 0.05). Dietary patterns, nutritional status, metabolic factors, and NAFLD are correlated. Furthermore, applying this correlation law can better manage NAFLD patients.

## 1. Introduction

Nonalcoholic fatty liver disease (NAFLD) is a chronic broad-spectrum clinical syndrome that starts from simple hepatic steatosis and can gradually develop into nonalcoholic steatohepatitis and finally develop into liver cirrhosis and even hepatocellular carcinoma [1, 2]. Studies have found that NAFLD patients tend to be obese, have insulin resistance, type 2 diabetes, dyslipidemia, hyperglycemia three hyperemia, and hypertension, which are also risk factors for cardiovascular diseases. NAFLD is the most common cause of liver function enzymatic abnormalities and chronic liver disease in western developed countries such as Europe and America. The prevalence of NAFLD in general adults is 20%–33%, with NASH and liver cirrhosis accounting for 10%–20% and 2%–3%, respectively. The prevalence of SFL in obese patients is 60%–90%, that of NASH is 20%–25%, that of cirrhosis is 2%–8%, and that of NAFLD in patients with type 2 diabetes mellitus and hyperlipidemia is 28%–55% and 27%–92%, respectively. With the global prevalence of obesity and metabolic syndrome, NAFLD in Asian countries has increased rapidly in the past 20 years with a trend of younger onset. The prevalence of NAFLD in adults in developed regions such as Shanghai, Guangzhou, and Hong Kong in China is about 15%. The annual incidence of NAFLD is 2% in Italy, 10% in Japan, and 3% in China. The annual incidence of NASH in women due to tamoxifen is estimated at 2% [3–5].

At present, there is still a lack of effective and safe drug treatment for NAFLD, and lifestyle intervention is still an important treatment for NAFLD patients, such as weight loss, a healthy diet, and increasing exercise [6]. Therefore, the prevention and treatment of NAFLD can be achieved by maintaining a healthy diet. For example, studies have shown that there is a positive correlation between the intake of foods rich in cholesterol, saturated fatty acids, or high fructose and the prevalence of NAFLD, such as sugary soft drinks and red meat [7, 8]. On the contrary, there was a negative correlation between n-3 polyunsaturated fatty acids and the prevalence of NAFLD.

Leptin is a polypeptide hormone encoded by the obesity gene, which plays an important role in the regulation of sugar and lipid metabolism in the liver. It acts on the hypothalamus and changes the dietary intake and energy consumption of the human body by regulating appetite increasing peptides and appetite inhibitory peptides. It is pointed out that it and its receptors are involved in the disorder of lipid metabolism in the liver. Leptin resistance is not only related to IR but also to the accumulation of fat in the liver. Adiponectin is an adipose hormone secreted mainly by adipocytes. Adiponectin levels are lower than normal in obesity, diabetes, and nonalcoholic fatty liver disease (NAFLD). Adiponectin has insulin sensitivity, which is related to insulin resistance and can reduce the secretion of tumor necrosis factor-*α* (TNF--*α*), fat accumulation, and inflammatory mediators in the liver [9]. Current studies have shown that there are two forms of adiponectin receptor-adiponectin 1 (adiponectin), which is mainly expressed in the skeletal muscle, and adiponectin receptor 2 (AdipoR2), which is mainly expressed in the liver. Some studies have shown that the level of adiponectin in patients with serum NAFLD is significantly lower than that in normal controls, suggesting that the decrease in serum adiponectin may be related to the pathogenesis of NAFLD [10]. More studies have shown that low serum adiponectin levels are associated with obesity and insulin resistance. According to the current research, adiponectin has been found for a long time, but as a metabolic factor in the diagnosis and treatment of type 2 diabetes, the significance of fatty liver, hypertension, coronary heart disease, and many other metabolic syndromes show that it has a broad research prospect [11, 12].

NAFLD is a metabolic stress liver injury closely related to insulin resistance and heredity. It is a common clinical cause of abnormal liver function or chronic liver disease. It is very common in patients with obesity, diabetes, hyperlipidemia, hypertension, hyperuricemia, and polycystic ovary syndrome. NAFLD is often very mild in its early stage, but it is very harmful. 80% of nonalcoholic fatty liver disease is simple fatty liver, most of which are found during physical examination, and the symptoms are relatively mild, because they are not specific, so they are ignored by people. If the disease is further aggravated, severe types of steatohepatitis can occur, and these patients will have chronic hepatitis manifestations such as liver pain, abdominal distension, fatigue, and poor appetite. This condition progresses to the intermediate stage of liver cirrhosis and hepatocellular carcinoma. The life expectancy of patients with nonalcoholic fatty liver disease is significantly shorter than that of ordinary people, and the main causes of death are cardiovascular disease and malignant tumors. Liver cancer and liver failure mainly occur in the stage of non-alcoholic steatohepatitis. In particular, among patients with liver cirrhosis, a survey has found that the prevalence rate can reach 15% among the general population in large and medium-sized cities. This kind of disease is becoming the first kind of liver disease in China, gradually replacing chronic hepatitis B and other liver inflammatory diseases. NAFLD is not a subhealth but a disease, which should be highly concern by the general public [13, 14].

In this study, we explore the correlation between nonalcoholic fatty liver disease (NAFLD) and dietary pattern, nutritional status, and metabolic factors, to provide a theoretical basis for the prevention and early intervention of NAFLD.

## 2. Materials and Methods

### 2.1. Study Design and Human Subject Collection

A total of 517 participants (200 males and 317 females) recruited in this study were gained from the health check center of The Ningbo Seventh Hospital, Ningbo, China, from September 2018 to August 2019. All subjects initially enrolled had complete health records on anthropometric examination, laboratory testing, and abdominal ultrasonography. NAFLD diagnosis was performed under the conditions of standard clinical evaluation following the Asia-Pacific Working Party criteria.

NAFLD can be diagnosed in those who have more than two of the following four findings of abdominal ultrasound abnormalities: (1) diffuse enhancement of liver near-field echo (bright liver), with stronger echo than kidney; (2) the structure of intrahepatic pipelines is not clear; (3) the far-field echo of the liver gradually decays; and (4) for patients with unexplained increases in serum alanine aminotransferase (ALT), if imaging studies suggest fatty liver and there are metabolic risk factors, NAFLD is the most likely cause of transaminase abnormalities.

The exclusion criteria were as follows: (1) alcohol consumption >140 g/week for males and >70 g/week for females; (2) history of viral hepatitis, drug-induced hepatitis, autoimmune hepatitis, and/or other forms of chronic liver disease, or currently on hepatotoxic medication; (3) body mass index (BMI) < 18.5 kg/m^2^; (4) missing dietary data; and (5) those who have changed their living habits within 5 years, including eating habits, drinking habits, smoking habits, exercise habits, and sleep habits. Written consent was assigned by all individual participants enrolled in this study.

### 2.2. Measurement of Dietary Intake

In this study, the semiquantitative food frequency questionnaire (FFQ) was used to evaluate the dietary intake data of participants. The food items in the questionnaire include seven options, which are 22 times a day, 1 time a day, 4–6 times a week, 2–3 times a week, 1 time a week, < 1 time a week, and almost no food according to the intake frequency. The beverage item includes 8 options, which are 24 cups per day, 2–3 cups per day, 1 cup per day, 4–6 cups per week, 2–3 cups per week, 1 cup per week, < 1 cup per week, and almost no drink according to the intake frequency. Participants must check their intake frequency of each food and beverage for one month in the abovementioned options. We calculate the daily average intake frequency of each food item of each participant according to the options checked by the participants and then calculate the daily average intake weight of each food item (g) in combination with the weight of each food item.

### 2.3. Ultrasonography and NAFLD Diagnosis

The hepatic ultrasonic examination was conducted by two trained ultrasonographers using a Toshiba Nemio 20 sonography machine (Toshiba, Tokyo, Japan) with a 3.5-MHz probe. NAFLD was diagnosed based on an ultrasound image with the evidence of hepatic steatosis after excluding significant alcohol consumption, hepatitis B/C, medication use, hereditary disorders, or any other definite liver damage factors.

### 2.4. Metabolic Syndrome Definition

The metabolic syndrome was defined according to the National Cholesterol Education Program (NCEP) Adult Treatment Panel III (ATP III) criteria [15, 16]. If at least three or more of the following five criteria are met, the metabolic syndrome is considered: (1) central obesity: waist circumference ≥90 cm in men and ≥80 cm in women; (2) hypertriglyceridemia: fasting TG ≥ 1.7 mmol/L; (3) low HDL-C: fasting HDL-C <1.03 mmol/L for men and <1.29 mmol/L for women; (4) hypertension: BP ≥130/85 mmHg and/or on anti-hypertensive drugs; and (5) hyperglycemia: FPG ≥5.6 mmol/L or previously diagnosed type 2 diabetes.

### 2.5. Statistical Analyses

Based on a cross-sectional study, the association between dietary pattern, nutritional status, metabolic factors level, and NAFLD were estimated. SPSS software package (version 22.0, IBM, USA) was employed for statistical analysis. The continuous variables were presented as mean ± standard deviation (SD) or median (interquartile range) as appropriate, whereas category variables were presented as number (%). Student's *t*-test and 2-test (for categorical variables) were used for between group comparisons flexibly according to conditions. To determine the correlation between dietary pattern, nutritional status, metabolic factors level, and NAFLD, Pearson correlation analysis was conducted. *P* < 0.05 (2-tailed test) was considered statistically significant.

## 3. Results

### 3.1. Characteristics of Subjects

A total of 517 eligible subjects (200 males and 317 females, mean age: 54.7 ± 16.7 years) were enrolled. Among them, 129 individuals (24.9%) were considered to be NAFLD. Moreover, there was no difference between the two groups in gender, BMI, blood pressure, aspartic acid, hypertension, diabetes, and smoking as shown in Table 1.

### 3.2. Associations between the Nutritional Status and NAFLD

In this study, the associations between nutritional status and NAFLD patients were explored. Our data indicated that BMI, body fat content, and waist-hip ratio were significantly different between the two groups (*P* < 0.05). However, no significant difference was observed in the body fat content between the two groups. Subsequently, we further analyzed the association between nutritional status and NAFLD. As shown in Tables 2 and 3 and Figure 1, the NAFLD patients have an obvious association with the waist-hip ratio.

### 3.3. The Association between Dietary Patterns and NAFLD

In this study, the associations between dietary patterns and NAFLD patients were explored. Our data indicated that dessert and fruit diets, healthy dietary patterns, animal food dietary patterns, and high salt diet mode were significant differences between the two groups (*P* < 0.05). However, no significant difference was observed in cereals and grain products diet mode between the two groups. Subsequently, we further analyzed the association between dietary patterns and NAFLD. As shown in Tables 3 and 4 and Figure 1, the NAFLD patients have an obvious association with dessert and fruit diet, healthy dietary pattern, animal food dietary pattern, and high salt diet mode.

### 3.4. Associations between Metabolic Factors and NAFLD

In this study, the associations between metabolic factors and NAFLD patients were explored. Our data indicated that triglyceride, uric acid, total cholesterol, and adiponectin were significantly different between the two groups (*P* < 0.05). However, no significant difference was observed in fasting blood glucose between the two groups. Subsequently, we further analyzed the association between metabolic factors and NAFLD. As shown in Tables 3 and 5 and Figure 1, the NAFLD patients have an obvious association with triglyceride, uric acid, and adiponectin.

## 4. Discussion

Nonalcoholic fatty liver disease has become the largest liver disease in China and one of the research hotspots of modern medicine. At present, the therapeutic drugs of Western medicine for NAFLD are still in the clinical trial stage, and there is a temporary lack of specific drugs. In recent years, more and more researchers have found that the occurrence and development of NAFLD are also closely related to the individual constitution of patients. Therefore, this study conducted a cross-sectional survey of NAFLD patients. The results included 517 patients to explore the correlation between NAFLD patients and dietary patterns, nutritional status, and metabolic indexes.

The ratio of BMI to actual weight and standard weight is a common index to evaluate the degree of obesity and further judge the nutritional status of the human body. The 2016 edition of the consensus of experts on medical nutrition treatment of overweight obesity in China defines those whose BMI level is greater than 24 kg/M2 as overweight, which is a manifestation of malnutrition. The WHO standard points out that the ratio of actual weight to standard weight is also one of the important indicators to evaluate the nutritional status. When it is greater than 10%, it can be defined as overweight [17, 18]. Among the 129 patients with NAFLD included in this study, the BMI level was more than 24 kg/m^2^, and the ratio of actual weight to standard weight was more than 10%. This suggests that more than 75% of patients in this study are overweight and obese, which indicates that malnutrition is common in NAFLD patients. The waist-hip ratio is an important index to judge central obesity. The average waist-hip ratio of NAFLD patients included in this study is 0.99 ± 0.86, which is higher than the normal level of waist-hip ratio of the general population in China (male: 0.81, female: 0.73). This suggests that NAFLD patients are mostly central obesity. Previous studies have found that obesity is an independent risk factor for NAFLD [19, 20], and weight loss is an important link in the intervention measures for NAFLD patients. Therefore, in the process of disease management of NAFLD patients, NAFLD patients should pay more attention to the relevant knowledge of diet management and weight control, to help patients do a better job in disease self-management.

This study found that NAFLD patients were positively correlated with TG and UA levels, and the TG level of NAFLD patients was significantly higher than that of the control group. Patients with high serum uric acid levels for a long time are more likely to suffer from damp and hot diseases such as gout stone deposition and gouty arthritis, so such patients have internal environment disorder. Therefore, for NAFLD patients, more attention should be paid to dietary management. It should be recommended that such patients pay special attention to eating less fat, sweet, greasy, and spicy products. At the same time, they should also limit the intake of shrimp and crab, fungi, bamboo shoots, soybean products, and other foods that are easy to lead to an increase in uric acid. In terms of monitoring and follow-up, NAFLD patients should monitor blood lipid, uric acid, and other indicators more closely than other physical fitness. In addition, this study also found that the average level of adiponectin in NAFLD patients was 2.26 ± 2.27 ug/L, in which NAFLD patients and serum adiponectin water. The results showed a strong positive correlation. Previous studies have shown that the more metabolic diseases are associated with hyperuricemia, hypertension, diabetes, and hyperlipidemia, the higher the serum adiponectin level is [21, 22]. This is consistent with our research results.

The results of this study found that the dietary patterns of sweets and fruits, a healthy diet, and animal food, all affect the prevalence of NAFLD through obesity or inflammation to varying degrees. At present, studies on dietary patterns and NAFLD both focus on the pathway of obesity, and EFA or PCA methods are used to extract the natural dietary patterns of the population. However, because the dietary pattern extracted by EFA or PCA mainly explains the variance of dietary data and does not contain the information on possible mediators of diet and disease, the dietary pattern extracted by EFA or PCA cannot become a predictor of disease in many cases. Animal food itself is a risk factor for the prevalence of NAFLD. At the same time, we found that the dietary pattern of sweets and fruits was positively correlated with the prevalence of NAFLD. In this dietary pattern, the intake of all kinds of fruits was high and speculated that the harmful effect of high fructose intake in fruits on NAFLD and the beneficial effect of antioxidants on NAFLD may offset each other. There may be differences in the content of fructose and antioxidants among various fruits, but because the population's preference for the intake of various fruits may be a whole, it is impossible to explore which kinds of fruits may be beneficial and which kinds of fruits may be harmful from this dietary pattern. To sum up, by discussing the key factors in the occurrence and development of NAFLD, combining these factors to build a purposeful dietary pattern (such as obesity and inflammatory dietary pattern), and then exploring the relationship between this dietary pattern and NAFLD, we can provide more information for the dietary prevention and treatment of NAFLD.

## 5. Conclusion

However, the limitations of our study must be discussed and documented in the paper. First, this was a cross-sectional observational study, so causality cannot be inferred. Second, this is a single-center study with a relatively small sample size, so it is necessary to increase the sample size to obtain more accurate experimental data to clarify our conclusions. Overall, despite the aforementioned limitations of this study, we first found that dietary patterns, nutritional status, metabolic factors, and NAFLD were associated. In addition, applying this correlation law may lead to better management of patients with NAFLD.

## Figures and Tables

**Figure 1:** Correlation scatter diagram.

**Table 1:** Clinical characteristics of two groups.

		NAFLD group (*n* = 129)	Non-NAFLD group (*n* = 388)	*P* value
*Sex*	Male	99 (76.7%)	144 (37.1%)	0.833
	Female	30 (23.3%)	73 (18.8%)	0.817
Age		55.5 ± 15.2	54.3 ± 17.1	0.087
BMI (kg/m^2^)		28.8 ± 4.3	25.9 ± 3.1	0.046
Systolic pressure (mmHg)		132.6 ± 16.4	127.1 ± 18.8	0.066
Diastolic pressure (mmHg)		80.3 ± 10.2	76.9 ± 10.6	0.081
Alanine aminotransferase		28.2 ± 17.2	19.6 ± 12.8	0.01
Aspartic acid		23.9 ± 9.4	21.6 ± 8.9	0.053
Triglyceride		2.78 ± 1.65	1.02 ± 0.32	0.03
Hypertension		39 (30.2%)	106 (27.3%)	0.096
Diabetes		8 (6.2%)	12 (3.1%)	0.062
Smoking		14 (10.9%)	59 (15.2%)	0.064

**Table 2:** Comparison of the nutritional status between the two groups $\left(\bar{x}\pm s\right)$.

	NAFLD group (*n* = 129)	Non-NAFLD group (*n* = 388)	*P* value
BMI (kg/m^2^)	28.8 ± 4.3	25.9 ± 3.1	0.046
Protein (%)	11.1 ± 1.86	12.3 ± 2.7	0.067
Body fat content (%)	27.57 ± 15.98	18.28 ± 3.9	0.035
Waist hip ratio (%)	0.99 ± 0.86	0.76 ± 0.05	0.013

Significant difference as *P* < 0.05.

**Table 3:** Univariate logistic regression analysis.

	*β*	SE	OR (95% CI)		*P*
Age	0.077	1.08	1.038	1.123	0.880
BMI (kg/m^2^)	−0.007	0.993	0.911	1.083	0.886
Systolic pressure (mmHg)	0.018	1.018	0.999	1.037	0.063
Diastolic pressure (mmHg)	0.050	1.051	1.018	1.085	0.062
Alanine aminotransferase	−0.049	0.953	0.488	1.860	0.887
Aspartic acid	0.953	2.594	1.255	5.358	0.810
Triglyceride	0.830	2.293	0.728	7.227	**0.006**
Hypertension	−0.052	0.949	0.103	8.705	0.963
Diabetes	1.369	3.93	0.538	28.704	0.177
Smoking	0.572	1.772	0.855	3.671	0.124
Protein (%)	0.018	1.018	0.484	2.141	0.962
Body fat content (%)	0.007	1.007	0.996	1.108	0.906
Waist hip ratio (%)	−0.011	0.989	0.985	0.993	**0.009**
Dessert and fruit diet	0.172	1.188	1.016	1.388	0.310
Healthy dietary pattern	−0.008	0.993	0.986	0.999	**0.027**
Animal food dietary pattern	0.126	1.134	1.034	1.244	**0.008**
High salt diet mode	0.000	1.000	1.000	1.001	**0.005**
Cereals and grain products diet mode	−0.088	0.916	0.820	1.023	0.120
FBG (mmol/L)	0.147	1.158	1.069	1.255	0.112
UA	−0.019	0.982	0.944	1.021	**0.010**
TC	0.008	1.008	0.929	1.094	0.850
Adiponectin	0.013	1.013	0.948	1.084	**0.005**

Significant difference as *P* < 0.05.

**Table 4:** Comparison of dietary patterns between the two groups $\left(\bar{x}\pm s\right)$.

	NAFLD group (*n* = 129)	Non-NAFLD group (*n* = 388)	*P* value
Dessert and fruit diet	36 (27.9%)	53 (13.7%)	**0.012**
Healthy dietary pattern	24 (18.6%)	188 (48.4%)	**0.008**
Animal food dietary pattern	33 (25.6%)	50 (12.9%)	**0.022**
High salt diet mode	47 (36.4%)	48 (12.4%)	**0.015**
Cereals and grain products diet mode	100 (77.5%)	305 (78.6%)	0.076

Significant difference as *P* < 0.05.

**Table 5:** Comparison of metabolic factors between the two groups $\left(\bar{x}\pm s\right)$.

	NAFLD group (*n* = 129)	Non-NAFLD group (*n* = 388)	*P* value
FBG (mmol/L)	5.81 ± 2.1	5.32 ± 1.49	0.066
TG (mmol/L)	2.78 ± 1.65	1.02 ± 0.32	0.03
UA	372.9 ± 90.2	316 ± 91	0.047
TC	5.08 ± 1.13	4.6 ± 0.89	0.032
Adiponectin	2.26 ± 2.27	1.8 ± 0.23	0.02

Significant difference as *P* < 0.05. FBG: fasting blood glucose; TG: triglyceride; UA: uric acid; TC: total cholesterol.

## Data Availability

The data supporting the findings of this study are available from the corresponding author.
